# Integrated Medical Care and the Continuous 4C Nursing Model to Improve Nursing Quality and Clinical Treatment of Patients with Acute Stroke: Based on a Retrospective Case-Control Study

**DOI:** 10.1155/2022/4810280

**Published:** 2022-06-06

**Authors:** Jing Zhang, Ling Ling Gu, Yan Xu, Bei Bei Zhao, Dan Li, ChunLing Xiao

**Affiliations:** ^1^School of Nursing and Midwifery, Jiangsu College of Nursing, Huai'an 223001, Jiangsu, China; ^2^Department of Emergency, Huai'an Second People's Hospital and The Affiliated Huai'an Hospital of Xuzhou Medical University, Huai'an, Jiangsu 223002, China

## Abstract

**Objective:**

This research paper is based on a retrospective case-control study for exploring the effects of medical nursing integration and the continuous 4C nursing model to improve the clinical treatment and nursing quality of patients with acute stroke.

**Method:**

For this purpose, a total of 313 patients with acute stroke, treated in our hospital from February 2020 to April 2021, were enrolled. They were divided into control and study groups with an even number of patients. The control group received integrated medical care number (*N* = 156), while the study group received integrated medical care and a continuous 4C nursing model (*N* = 157). In integrated medical care, the general data, self-nursing ability, degree of neurological impairment, Fugl–Meyer Assessment (FMA) score, Barthel index score, and quality of life score were compared between the two groups.

**Result:**

The self-nursing concept, self-nursing responsibility, self-nursing skills, health knowledge, and total score of the patients in the study group were higher than those in the control group (*P* < 0.05). The neurological function scores of the study group were lower than those of the control group at 1, 3, and 6 months after discharge (*P* < 0.05). The scores of the study group were higher than those of the control group at 1, 3, and 6 months after discharge (*P* < 0.05). The Barthel index score of the study group was higher than that of the control group at 1, 3, and 6 months after discharge. The scores of physical function, psychological function, social function, and health self-cognition in the study group were lower than those in the control group (*P* < 0.05).

**Conclusion:**

The application of integrated medical care and the continuous 4C nursing model for patients with acute stroke is beneficial to enhance the degree of neurological impairment of stroke patients, improve activities of daily life and motor function, and facilitate patients' quality of life. It is helpful to strengthen the attitude and feeling of cooperation between doctors and nurses, promote cooperation between doctors and nurses, reduce the defects of nursing work, heighten the quality of nursing, and achieve the requirement and goal of effectively promoting high-quality nursing.

## 1. Introduction

Generally speaking, stroke refers to the acute disturbance of cerebral blood circulation caused by cerebrovascular diseases caused by various factors. It is characterized by symptoms of one-time or permanent brain dysfunction [1]. Results of the past decades show that the annual death toll from stroke is more than 2 million. However, the annual death rate is increasing at 8.7% [1]. According to the survey of the World Health Organization (WHO), the incidence of stroke in China ranks first in the world, which is twice as high as in the United States. Stroke not only has a high fatality rate but also has the characteristics of high disability and a high recurrence rate. It is a serious threat to the quality of life of the patient [2]. Stroke management has been used as the main curing method for stroke patients in many countries. However, developing a set of nursing quality indicators matched with stroke treatment is particularly important [3]. Some studies have shown that hospitalization can improve the prognosis of stroke patients. In addition, the recently published guidelines for stroke nursing assessment also recommend the direct or indirect application of quality indicators to assess the quality of stroke care [4]. In recent years, many studies have been devoted to improving the nursing quality index of stroke, so that it can give full play to the role of supervision and guidance in quality control and provide a basis for continuous nursing quality [4]. At present, the nursing quality index of stroke monitoring, as the quality control standard of a hospital, has been established in Europe, but there is no consensus on the content and method of the stroke nursing quality index [4].The research in the field of the stroke nursing quality index in China is still in its infancy. How to proceed from the reality of nursing quality management and learn from various advanced management methods and means to establish a scientific stroke nursing quality system needs in-depth research [5].

In the whole process of health services, the harmonious relationship between doctors and nurses has a direct impact on the outcome of patients [3]. Integrated health care does not only mean that doctors and nurses work together but also it is a process in which doctors and nurses work independently, collaborate and share information and responsibilities. Diagnosis and treatment, health education, and rehabilitation programs are jointly formulated by doctors, nurses, and patients after full communication. They assist each other in the decision-making and implementation process [6]. Integrated medical care builds a bridge between doctors and nurses. It makes the communication and cooperation between doctors and nurses more efficient. In the beginning, the relationship between doctors and nurses was dominated by doctors, and nurses carried out the relationship subordinately. Now, it has gradually changed to active communication, cooperation, and coleadership [7]. In the meanwhile, this model makes the communication channels between doctors and nurses more unobstructed and effective and can quickly realize the sharing of patient-related information, so that both doctors and nurses can have a more comprehensive understanding of the needs and patients' conditions. It is beneficial to make correct clinical medical and clinical nursing rehabilitation decisions to improve the overall service quality of health care [7, 8]. The 4 C continuous nursing model is developed based on the Omaha system, including four “C”: comprehensiveness, cooperation, coordination, and continuity of the nursing service process [9]. Comprehensiveness refers to the assessment of physical, psychological, health behavior, and social environmental health problems when patients are discharged from the hospital and enter their daily life activities and foresee their health needs [10]. Cooperation means strengthening cooperation between patients and health care workers. Coordination means multidisciplinary docking and coordination. Continuity refers to the continuous and regular provision of nursing follow-up services after discharge. In the past, it is often reported that the comprehensive nursing model and continuous 4C nursing model are used alone in the nursing of acute stroke, but there are a few reports of the combination of the two. In this study, a retrospective case-control study was conducted to explore the effect of integrated medical treatment and the continuous 4C nursing model on improving the clinical treatment and nursing quality of patients with acute stroke. It is beneficial to enhance the degree of neurological impairment of stroke patients, improve activities of daily life and motor function, and facilitate patients' quality of life. It is helpful to strengthen the attitude and feeling of cooperation between doctors and nurses, promote cooperation between doctors and nurses, reduce the defects of nursing work, heighten the quality of nursing, and achieve the requirement and goal of effectively promoting high-quality nursing. The rest of the paper is organized as follows: the following section will explain the patients and methods used in the study. It will be followed by results and discussion. Finally, the study will be concluded in the last section.

## 2. Patients and Methods

In this section, the details of stroke-diagnosed patients along with the methods and tools used for the diagnosis will be explained.

### 2.1. Demographic Data

A total of 313 patients with acute stroke treated in our hospital from February 2020 to April 2021 were enrolled. They were divided into control and study groups with an even number of patients. The control group received integrated medical care (*N* = 156), and the study group received integrated medical care and a continuous 4C nursing model (*N* = 157). In the control group, the age ranged between 43 and 74 years. While in the study group, the age ranged between 44 and 76 years. This study was approved by the Medical Ethics Association of our hospital, and all patients signed informed consent, which is in line with the rules of the Helsinki Declaration (revised in 2013).

#### 2.1.1. Selection Criteria

The selection criteria for the patients are described as follows: according to the diagnostic criteria of cerebral hemorrhage and cerebral infarction in the diagnostic essentials of various cerebrovascular diseases adopted by the Chinese Medical Association in the fourth National Cerebrovascular Disease Academic Conference and combined with CT or MRI examination, acute stroke was diagnosed.

The vital signs were stable, and there was no obvious disturbance of consciousness after treatment.

The age ranged between 20 and 85 years. Four patients agreed to accept the follow-up for 6 months and be able to accept and answer telephone calls.

#### 2.1.2. Exclusion Criteria

The exclusion criteria for the patients are described as follows: patients with severe diseases of the circulatory system, digestive system, respiratory system, endocrine system, or malignant tumors that seriously affect the quality of life.

Patients with severe aphasia, cognitive impairment or dementia, mental illness, or unable to cooperate with researchers.

Those who have undergone clinical trials within 3 months and take observation drugs.

Those with a history of mental illness and drug abuse lead to the aggravation of depression.

Unable to cooperate or unwilling to cooperate.

### 2.2. Nursing Methods

The different nursing methods and tools used are explained as follows.

#### 2.2.1. Establishment of the Integrated Nursing Group

The control group received integrated medical care and adopted the integrated clinical nursing model to construct a stroke specialist medical nursing unit. In the multidisciplinary team of integrated doctors and nurses, the responsibility of treatment, nursing, rehabilitation, health education, standardized integrated medical, and nursing services were provided for stroke patients. The integrated diagnosis and nursing group is composed of experienced clinical neurologists, trained professional stroke nurses, and rehabilitation specialists. According to the professional titles and energy levels of doctors and nurses, they were divided into three integrated medical and nursing groups; each one of them was in charge of 1–5 beds. The chief physician serves as the medical team leader of the nursing group, and the nurses at N3 levels serve as the nursing team leader of the nursing group. It includes physicians, N2, and N1 nurses. The members of the group received regular details of training on knowledge related to cerebrovascular diseases, including nursing guidelines for stroke treatment, diagnosis, stroke scale training, and stroke rehabilitation training, so that the knowledge of the members of the medical and nursing integration group was constantly updated. At the same time, doctors and nurses jointly completed a comprehensive assessment of the physical health, physiological status, social support, and emotional status of stroke patients, including patients' self-care ability, physical activity ability, language, swallowing, and cognitive ability.

#### 2.2.2. Establishment of the Integrated Medical and Nursing System

Doctors and nurses have made joint rounds. The original nurse scheduling model has also been changed. For nurses participating in ward rounds, the schedule is marked with a1, a2, b2, b2, C1, and c2. The A, B, and C represent three nursing groups, respectively. A1 nurses are in charge of the first eight beds of the first consultation. Similarly, A2 nurses are in charge of the last eight beds of the first consultation and nursing group. Nurses follow the doctors of the same diagnosis and nursing group. They are jointly responsible for the treatment, nursing, and rehabilitation of the patients. During ward rounds, the health care room uses a standardized way of communication, involving every link of information communication, showing what is happening to the patient, what are the causes, its impacts, and solution to the problem. In the ward rounds, the doctor put forward the nursing requirements and suggestions to the existing problem for the patients. They also evaluate and give feedback to the dialectical nursing group. The nurses accurately follow the doctor's orders, closely observe the changes in patients' condition, carry out in-depth communication with doctors on medical history and formulate a more effective diagnosis, treatment, and nursing methods, and strengthen communication and assistance between doctors and nurses. However, the nursing and rehabilitation programs should be adjusted with time according to the changes of the disease. For difficult cases, the diagnosis and nursing team regularly carry out multidisciplinary case seminars to put forward the existing problems of the patients and actively solve them. To ensure the quality of ward rounds, the department uniformly distributes ward round notebooks to nurses, asking the nurses to listen carefully to the doctors' requirements, take the initiative to participate in the process of ward rounds, and put forward reasonable opinions and suggestions on the nursing care of the disease. They have to conscientiously take notes on ward rounds and hand them over to the nursing leader of each group before leaving work. The head nurse summarizes the data on the same day and gave timely feedback on the changes in the treatment, nursing, and rehabilitation of the patients. The head nurse regularly inspected and reviewed the notes of the nurses' rounds.

The study group accepted the integrated medical care and continuous 4C nursing model. The integrated medical care was the same as in the control group. Meanwhile, the following continuous 4C nursing model was adopted: nursing intervention was carried out around the “comprehensive” and “cooperative” of the 4C continuous nursing model. The results are as follows.

After the patient is admitted to the hospital, the competent nurse will introduce the ward environment and evaluate the problems faced by the patient in the four areas: environment, psychosocial, physiology, and health. The attention of the attending physician is important in popularizing the science of acute stroke.

Before being discharged, the patient files of nursing graduate students are registered. It includes general information (name, sex, personality, age, educational background, occupation, income, type of health insurance, religion, etc.), treatment, mode of operation, assessment of physical needs, cognition of disease, psychological needs, social support, and others, and investigation of quality of life and self-care ability. Also, a communication line, such as, a WeChat account and mobile phone number, between the patient and hospital is also being made.

The training of patients or their family members related to acute stroke should be completed by specialist nurses.

Psychological counselors and dietitians evaluate the psychological and nutritional status of patients, marked with red for patients who may have negative psychological reactions and blue for patients with malnutrition. Psychological counseling and nutritional guidance were given to the patients according to their conditions. After discharge, follow-up intervention was carried out around “coordination” and “continuity” in the 4C continuous nursing model.

4C team members push relevant content on the communication line regularly according to the plan. Patients learn on time, encourage family members to participate in the learning process of patients, and supervise the patients.

Intermittently, a follow-up has to be arranged with the patients regularly on the video communication line. We need to formulate the next intervention goal and plan according to the patients' physical, psychological, and nutritional conditions and let the patients make comments and opinions at the end of each survey.

Patients are invited to participate in activities such as “sunshine sleep” and “patient fraternity” held in each period to encourage patients to restore their own experience and regain their confidence.

Regular intragroup interactive questions and answers, according to the common questions of multiple patients during each video follow-up, after being answered, were collected again, and sent to the group to share. For other convalescent questions raised by patients that are not related to this study, the researchers consult clinically experienced doctors or nurses before answering them.

### 2.3. Observation Index

The observation index of this research is as follows.

#### 2.3.1. General information

Statistics of the general data and indicators of the two groups of patients, including patients' age, occupation, marital status, education level, and concomitant diseases, were compared.

#### 2.3.2. Self-Care Ability

In the late 1970s, the Kearney research group of American scholars developed the scale based on Orem's self-care theory [11], involving four dimensions as follows: self-care concept (entry 1–8), self-care responsibility (entry 9–14), self-care skills (entry 15–26), and health knowledge level (entry 27–43). Cronbach's *α* of the scale is 0.87. Using the Likert5 grade scoring method, 11 items were scored in reverse, and the highest score was less or equal to 172. The higher score indicates the stronger self-nursing ability of the patients.

#### 2.3.3. Neurological Deficit Score

The neurological deficit was assessed by the Chinese Stroke patients' Neurological Deficit Rating Scale (CSS) [12]. It included myodynamia, speech disorder, mental disorder, walking ability, hemiplegia, and eyeball disorder. The total score was 45. The higher score indicates the seriousness of the neurological impairment.

#### 2.3.4. Limb Motor Function

The score of the Fugl–Meyer Assessment (FMA) rating scale of limb motor function was assessed [13]. The points were divided as follows: 50 points for severe dyskinesia, 51–84 points for obvious dyskinesia, 85–95 points for moderate dyskinesia, and 96–99 points for mild dyskinesia.

#### 2.3.5. Barthel Index

The Barthel index [14] was used to evaluate the ability of daily life before and after intervention. The total score was 100. The higher score indicates stronger ability of daily life.

#### 2.3.6. Quality of Life Scale

The quality of life scale [15] consists of four subscales. It includes physical, psychological, social, and health self-awareness, with a total of 29 items. Cronbach's *α* coefficient of the scale is 0.79 to 0.91. The scale was scored by 1–5 grades. A lower score indicates a higher rate of satisfaction.

### 2.4. Statistical Analysis

SPSS21.0 was used for data analysis. Mean, standard deviation, median, quartile spacing, and constituent ratio were used for statistical description. The baseline data were analyzed by *χ*^2^ test and two-sample independent *t*-tests. If the data type belongs to measurement data and accords with normality, repeated measurement analysis of variance or two independent samples *t*-test, nonnormality data, nonparametric test, chi-square test, and nonparametric test are used. *P* < 0.05 indicates that the difference is statistically significant.

## 3. Results

The results extracted from this study are as follows:

### 3.1. Comparison of General Demographic Data

First of all, we compared the general data of the two groups; there was no significant difference in age, occupation, marital status, education level, concomitant disease, and other general data between the two groups (*P* > 0.05). All the data are shown in Table 1.

### 3.2. Comparison of the Self-Nursing Ability

Secondly, we compared the self-nursing ability of the two groups, and there was no significant difference between the two groups (*P* > 0.05). The scores of the self-nursing concept, self-nursing responsibility, self-nursing skills, health knowledge, and total score in the study group were significantly higher than those of the control group (*P* < 0.05). All the results are shown in Table 2.

### 3.3. Comparison of the Degree of Neurological Impairment

Then, we compared the degree of neurological impairment between the two groups. Before nursing, there was no significant difference between the two groups (*P* > 0.05). The score of neurological impairment in the study group was lower than that of the control group at 1, 3, and 6 months after discharge. The difference was statistically significant (*P* < 0.05). All the results are shown in Table 3.

### 3.4. FMA Score Comparison

Next, we compared the FMA scores of the two groups. There was no significant difference between the two groups before nursing, but after nursing, the FMA scores of the two groups increased. The scores of the study group at 1, 3, and 6 months after discharge were higher than those of the control group. The difference was statistically significant. All the results are shown in Table 4.

### 3.5. Comparison of Barthel Index

Next, we compared the Barthel index scores of the two groups. There was no significant difference between the two groups before nursing, but after nursing, the Barthel index scores of the two groups increased. The score of the study group at 1, 3, and 6 months after discharge was higher than that of the control group. The difference was statistically significant. All the results are shown in Table 5.

### 3.6. Comparison of the Quality of Life Scores

Finally, we compared the scores of the quality of life between the two groups. Before nursing, there was no significant difference between the two groups (*P* > 0.05). The scores of physiological function, psychological function, social function, and health self-cognition in the study group were lower than those of the control group. The difference was statistically significant (*P* < 0.05). All the results are shown in Table 6.

## 4. Discussion

Stroke generally refers to the local or diffuse brain function damage caused by persistent cerebral ischemia or hypoxia, which is caused by insufficient blood supply or interruption of blood flow in the corresponding brain functional areas promoted by cerebral vascular occlusion or cerebral vascular rupture [16, 17]. Stroke has the characteristics of high disability, fatality, high recurrence, and a long rehabilitation cycle. According to statistics, 69% of stroke patients are over 65 years of age. With the aging of the population, the incidence of stroke is increasing day by day. The complications caused by stroke, such as disturbance of consciousness, hemiplegia, and loss of speech function, seriously affect the quality of life of patients and become an important threat to the disability of the elderly population. It has also brought great economic and mental pressure to the patient's family and medical unit [18]. Stroke recurrence early warning and continuous nursing service are important forms to reduce the risk of stroke and the rate of death and disability and to promote rapid rehabilitation [18]. At present, the main body of continuous service for stroke patients is mainly nurses in medical units, but due to the increasing number of stroke patients year by year, continuous service has greatly increased the burden on nurses. They cannot be motivated. In addition, the quality of nurses is uneven; lack of in-depth understanding of continuous nursing, which cannot provide quality services for stroke patients, affects the functional recovery of stroke patients. Therefore, there is an urgent need for an efficient continuous nursing model for stroke patients [19].

As early as 1947, a report of the American Nursing Association first mentioned the model of continuous care but did not elaborate it in detail. In 2003, the American Geriatric Association defined the model: continuous care refers to the continuation of patients from the hospital to the family through a series of action designs to ensure that the patients receive different levels of collaborative and continuous care in different health care places to prevent or reduce the deterioration of patients' health status [20]. The more common continuous nursing models include the discharge planning model, transitional nursing model, and case management model. From admission to discharge, a linked health management network is formed by inpatient hospitals, community clinics, and family doctors to achieve layer-to-layer linkage and continuous care at all levels to ensure that patients can receive better nursing services after discharge. Professionally trained nurses, community personnel, and social workers help patients carry out their health management and make appointments for family doctors and family visits, suggesting that patients can record their health changes dynamically [21]. The continuous nursing model guided by senior practical nurses will develop rapidly in the next decade and will be the mainstream of continuous nursing. Through the guidance of senior practising nurses, to assist patients to transfer from the hospital to the family or community, patients through the mobile network to maintain contact with senior practice nurses, timely access to out-of-hospital health care. After the continuous exploration of scholars, multidisciplinary teams are encouraged to join the continuous nursing team guided by senior practical nurses to provide professional nursing services for patients [22]. In 2001, some scholars built a conceptual model of continuous nursing based on six dimensions, and later other scholars supplemented the core elements, which provided a good idea for the development of continuous nursing. At present, a variety of continuous nursing models abroad have passed the test of practice, such as the continuous nursing intervention model, APN continuous nursing model, elderly resource model for taking care of the elderly, and guided nursing model.

This study found that the self-nursing concept, self-nursing responsibility, self-nursing skills, health knowledge, and total score of the patients in the study group were higher than those in the control group (*P* < 0.05). The neurological function scores of the study group were lower than those of the control group at 1, 3, and 6 months after discharge (*P* < 0.05). The scores of the study group were higher than those of the control group at 1, 3, and 6 months after discharge (*P* < 0.05). The Barthel index score of the study group was higher than that of the control group at 1, 3, and 6 months after discharge. The scores of physical function, psychological function, social function, and health self-cognition in the study group were lower than those in the control group (*P* < 0.05). The reasons are as follows: with the formation of the new medical model, disease treatment, and nursing are no longer the only focus of medical services, but to provide comprehensive medical services for patients, emphasizing the provision of humanized and individualized continuous full-process medical services and providing health services for patients [23, 24]. Nurses can not only correctly understand doctors' orders but also execute them timely and accurately. They have professional clinical skills that they are familiar with in marriage; have excellent first aid knowledge and can make an emergency response in emergencies; have a keen ability to observe the disease and report to the doctor in time; and have a strong ability to communicate with patients and their families. Through communication with patients and their families in nursing work, we can put forward opinions and suggestions on diagnosis and treatment according to nursing experience. In the meanwhile, nurses also hope that doctors can do the following: clear diagnosis, proper treatment, planned work; accurate, concise, timely, specific, and centralized doctor's orders and actively cooperate with nurses in psychological counseling and necessary explanation; doctors respect and affirm the work of nurses, establish, actively maintain the prestige of nurses in front of patients and family members, and actively help nurses to improve their medical knowledge and skillfulness. The significance and effect of the integrated work model of health care can be divided into two aspects: the effect on health care and the effect on patients [24]. Thus, it can be seen that integrated medical care can promote the harmonious relationship between doctors and nurses, promote cooperative behavior between doctors and nurses, and expand the connotation of nursing work, so as to achieve high-quality and efficient medical and health services. The integration of health care and nursing is helpful for doctors and nurses to agree on the changes of patients' condition, treatment plan, nursing plan, and rehabilitation plan, so as to effectively reduce and avoid the occurrence of subjective judgment or lack of understanding of patients' condition and diagnosis and treatment plan caused by poor communication between doctors and nurses [24]. In addition, nurses put forward to doctors what they do not understand or have doubts about, correctly understand and grasp the main points of patients' treatment and nursing, and timely and accurately provide doctors with information on patients' condition changes, nursing effects, and psychological status, which can better implement correct clinical decisions, achieve optimal cooperation, and complementarity between doctors and nurses, and thus, improve the job satisfaction of doctors and nurses [25].

On the other hand, through the implementation of integrated medical care, patients can also benefit from it. He et al. found that the mortality rate of AIDS patients in hospitals with good health care integration cooperation is 0.5% lower than that in general hospitals through research on hospitals with better health care integration cooperation [26]. Concomitantly, the implementation of integrated medical care in the operating room can make communication between the medical staff and the patients more positive, effectively improve the anxiety and depression of the patients, and enhance the matching degree of the patients. Moreover, integrated medical care can reduce hospital costs and patients' medical expenses, improve patients' clinical outcomes, strengthen medical care, nursing quality, and service efficiency, and reduce tensions and conflicts between doctors and nurses, fostering the satisfaction of patients and their families [27]. In addition, the quality of health care cooperation behavior has a direct impact on medical quality, health care relationship, patient health outcome, and patient satisfaction. The joint rounds of doctors and nurses and nurses' participation in the whole process of medical nursing rehabilitation decision-making can enable nurses to better understand the progress of patients' condition and the changes of treatment and rehabilitation, effectively reduce errors and risk accidents in medical care, and make nursing for patients more personalized more in line with the treatment plans and rehabilitation goals of doctors and recovered patients and can also improve the overall medical quality. As a result, the job satisfaction and sense of professional value of medical staff are improved [28]. Integrated medical care requires nurses to integrate the participation of doctors and patients into clinical nursing work, such as nursing procedures and health education, and to jointly formulate diagnosis and treatment plans through benign communication and good cooperation to achieve the complementarity of specialized knowledge and professional skills between doctors and nurses, and patients and caregivers receive consistent and standardized scientific rehabilitation guidance and assistance from different aspects, which provides a good treatment and nursing environment for patients [29]. Some studies have proposed that integrated medical care can promote the professional development of nurses, and it can also be used as an effective supplementary way and form of nursing continuing education project [30].

## 5. Conclusion

To sum up, the application of integrated medical treatment and the continuous 4C nursing model in patients with acute stroke is beneficial to improve the degree of neurological impairment, activities of daily living, and motor function and improve the quality of life of patients with stroke. It helps to strengthen the attitude and feeling of cooperation between doctors and nurses, promote cooperation between doctors and nurses, reduce the defects of nursing work, improve nursing quality, and achieve the requirements and goals of effectively promoting high-quality nursing.

## Figures and Tables

**Table 1:** Comparison of general demographic data.

Group	Control (*n* = 156)	Study (*n* = 157)	*t*/*χ*^2^	*P*
Age (years)	56.81 ± 3.91	56.83 ± 3.36	0.048	0.961
Gender (male/female)	74/82	78/79	0.158	0.691

Career				
On the job	47 (30.17%)	48 (30.57%)	1.912	0.384
Retired	70 (44.87%)	60 (38.22%)		
Others	39 (25.00%)	49 (31.21%)		

*Marital status*				
Married	68 (43.59%)	63 (40.13%)	2.625	0.269
Not married	23 (14.74%)	16 (10.19%)		
Divorced/widowed	65 (41.67%)	78 (49.68%)		

*Degree of education*				
Primary school	31 (19.87%)	23 (14.65%)	2.686	0.442
Junior middle school	31 (19.87%)	28 (17.83%)		
High school	67 (42.95%)	70 (44.59%)		
Senior high school and above	27 (17.31%)	36 (22.93%)		

*Concomitant disease*				
1	31 (19.87%)	32 (20.38%)	0.412	0.813
2	27 (17.31%)	23 (14.65%)		
≥3	98 (62.82%)	102 (64.97%)		

**Table 2:** Comparison of the self-nursing ability ($\bar{x}$ ± *s*).

Group	*N*	Self-care concept	Sense of responsibility for self-care	Self-nursing skills	Health knowledge level	Total score
Control	156	19.86 ± 4.67	16.79 ± 4.25	18.97 ± 4.66	38.91 ± 5.23	96.81 ± 8.52
Study	157	23.85 ± 3.31	25.83 ± 3.31	23.86 ± 4.33	45.71 ± 3.44	124.85 ± 9.67
*t*		8.724	21.001	9.617	13.597	27.121
*P*		0.001	0.001	0.001	0.001	0.001

**Table 3:** Comparison of the degree of neurological impairment.

Group	*N*	Before nursing	Discharge	1 month after discharge	3 months after discharge	6 months after discharge
Control	156	26.83 ± 3.11	22.83 ± 2.46^a^	20.48 ± 3.30^ab^	16.79 ± 2.22^abc^	14.82 ± 2.43^abcd^
Study	157	26.85 ± 3.54	20.81 ± 1.64^a^	17.84 ± 1.35^ab^	14.93 ± 1.34^abc^	12.48 ± 1.44^abcd^
*t*		0.053	8.552	9.273	8.980	10.371
*P*		0.957	0.001	0.001	0.001	0.001

*Note.* Compared with before nursing, aP < 0.05; compared with discharge, bP < 0.05; compared with 1 month after discharge, cP < 0.05; compared with 3 month after discharge, dP < 0.05.

**Table 4:** FMA score comparison.

Group	*N*	Before nursing	Discharge	1 month after discharge	3 months after discharge	6 months after discharge
Control	156	61.93 ± 3.45	63.31 ± 1.46^a^	64.81 ± 3.11^ab^	68.83 ± 3.18^abc^	73.83 ± 3.67^abcd^
Study	157	61.96 ± 4.31	65.93 ± 4.11^a^	67.84 ± 4.31^ab^	73.58 ± 3.31^abc^	80.83 ± 3.15^abcd^
*t*		0.067	7.505	7.128	12.945	18.110
*P*		0.945	0.001	0.001	0.001	0.001

*Note.* Compared with before nursing, aP < 0.05; compared with discharge, bP < 0.05; compared with 1 month after discharge, cP < 0.05; compared with 3 months after discharge, dP < 0.05.

**Table 5:** Comparison of the Barthel index.

Group	*N*	Before nursing	Discharge	1 month after discharge	3 months after discharge	6 months after discharge
Control	156	33.55 ± 3.75	46.54 ± 3.33^a^	54.34 ± 5.56^ab^	78.77 ± 4.32^abc^	88.42 ± 3.87^abcd^
Study	157	33.31 ± 3.42	58.42 ± 4.77^a^	65.65 ± 3.42^ab^	84.55 ± 5.67^abc^	98.67 ± 4.86^abcd^
*t*		0.591	25.533	21.690	10.139	20.632
*P*		0.554	0.001	0.001	0.001	0.001

*Note.* Compared with before nursing, aP < 0.05; compared with discharge, bP < 0.05; compared with 1 month after discharge, cP < 0.05; compared with 3 months after discharge, dP < 0.05.

**Table 6:** Comparison of the quality of life scores.

Group	*N*	Physiological function		Psychological function		Social function		Healthy self-cognition	
		Before nursing	After nursing	Before nursing	After nursing	Before nursing	After nursing	Before nursing	After nursing
Control	156	14.84 ± 4.64	13.53 ± 2.65^a^	16.44 ± 3.66	14.95 ± 4.17^a^	18.87 ± 3.34	16.92 ± 2.85^a^	15.86 ± 3.43	13.85 ± 1.71^a^
Study	157	14.53 ± 4.44	12.16 ± 0.44^b^	16.42 ± 3.86	12.86 ± 1.65^b^	18.81 ± 3.66	12.84 ± 3.97^b^	15.94 ± 3.65	10.7 ± 2.87^b^
*t*		0.603	6.389	0.047	5.873	0.154	10.438	0.199	2.972
*P*		0.546	0.001	0.962	0.001	0.879	0.001	0.841	0.003

*Note.* The control group before and after nursing, aP < 0.05; the study group before and after nursing, bP < 0.05.

## Data Availability

The datasets used and analyzed during the current study are available from the corresponding author upon reasonable request.
